The article "Automatic Detection and Classification of Epileptic Seizures in Patients with Liver Cirrhosis and Overlapping Hev Infection Based on Deep Multimodal Fusion Technology" was retracted in 2023. Reasons: signs of a paper mill; compromised peer review; unreliable results or conclusions.

# Automatic Detection and Classification of Epileptic Seizures in Patients with Liver Cirrhosis and Overlapping Hev Infection Based on Deep Multimodal Fusion Technology

**DOI:** 10.1155/2022/3176134

**Published:** 2022-08-31

**Authors:** Jianan Yu, Rui Min, Yun Yu, Xiaorui Hu, Xiandong Fu, Nannan Chi

**Affiliations:** ^1^Department of Neurology, The First Affiliated Hospital of Jiamusi University, Jiamusi 154000, Heilongjiang, China; ^2^Emergency Department, The First Affiliated Hospital of Jiamusi University, Jiamusi 154000, Heilongjiang, China; ^3^Department of Medical Education, The First Affiliated Hospital of Jiamusi University, Jiamusi 154000, Heilongjiang, China; ^4^Department of Psychiatry, The First Affiliated Hospital of Harbin Medical University, Harbin 150000, Heilongjiang, China; ^5^Department of General Surgery, The First Affiliated Hospital of Jiamusi University, Jiamusi 154000, Heilongjiang, China; ^6^Digestive Department, The First Affiliated Hospital of Jiamusi University, Jiamusi 154000, Heilongjiang, China

## Abstract

Liver cirrhosis is a clinical chronic developmental liver disease, which is caused by long-term or repeated effects of liver dysfunction, and there are more and more cases of epileptic seizures in patients with liver cirrhosis and HEV infection. This article aims to study how to analyze epileptic seizures in patients with liver cirrhosis and overlapping HEV infection based on deep multimodal fusion technology. This article proposes a deep learning neural network algorithm based on deep multimodal fusion technology, and how to use this algorithm to automatically detect and classify epileptic seizures. The data in the experiment in this article show that the prevalence of epilepsy accounts for 1% of the world's population, about 56.7 million people, and 1 in 25 people may have an epileptic seizure at some time in their lives, and in each person's life, the probability of seizures due to various reasons is 10%. In 2016, the proportion of males with cirrhosis reached 16%, females reached 8%, and males were 8% higher than females, which is a full double. The test results show that with the increase in patients with cirrhosis and overlapping HEV infection, the frequency of epileptic seizures is also getting higher and higher, indicating that the frequency of epileptic seizures has been increased in patients with cirrhosis and overlapping HEV infection. Therefore, it is imperative to analyze the epileptic seizures of patients with liver cirrhosis and overlapping HEV infection based on deep multimodal fusion technology.

## 1. Introduction

Epilepsy is a disease that affects the overall health of an individual. With the transformation of medical models and the development of cognitive neuroscience, people have realized that epilepsy, like other brain diseases in humans, has the problem of brain dysfunction, which is accompanied by neurobiological, cognitive, and psychological changes, and there are complex cognitive impairments. There are obvious challenges in the life situation of patients with epilepsy, because they not only have the fear of repeated epilepsy and uncertainty, they need to face long-term epilepsy treatment, but also have limited daily activities, decline in social function, family conflicts, stigma, and accompanying mental illnesses such as depression and anxiety.

In recent years, with the development of medical technology, the treatment of epilepsy has made new progress in the field of epilepsy, but about one-third of the patients with epilepsy are still very low in the efficacy of drug treatment. Epilepsy is a chronic disease in which sudden, abnormal discharge of brain neurons can cause transient brain dysfunction. Treatment mainly depends on drugs. Cirrhosis is a common clinical chronic progressive liver disease, diffuse liver damage caused by long-term or repeated actions of one or more causes, and hence it is of great significance to analyze the seizures of patients with liver cirrhosis and overlapping HEV infection based on deep multimodal fusion technology.

The rapid development of Internet technology has had a great impact on people's lives, and in particular, the rapid development of mobile Internet in recent years has made it very convenient for people to interact with information. Cuppens found that due to the cumbersome way to monitor epileptic seizures using standard methods of EEG monitoring, night-time home monitoring of children with epilepsy is usually not feasible. He proposed a method for detecting hyperkinetic epilepsy based on accelerometers connected to the extremities, which is from the acceleration signal; multiple features based on time, frequency, and wavelet are extracted, and after determining the feature with the highest discriminative power, the motion events are divided into epileptic and non-epilepsy motion, and this classification is only based on the non-parametric estimation of the probability density function of normal motion. This method enables the construction of patient-specific models to classify exercise data without the need for rarely available seizure data [1, 2]. If during the testing phase, the probability of a data point is below the threshold, the event is considered to be a seizure; otherwise, it is considered to be a normal night movement event. The average performance of 7 patients gave a sensitivity of 95.24% and a positive predictive value of 60 [3]. Vespa found that traumatic brain injury can cause continuous interruption of brain metabolism, which has not yet been mechanically defined. Early post-traumatic seizures are a potential mechanism of metabolic crisis, and therefore may be a treatment target. It is hypothesized that seizures and false periodic discharges may be mechanistically related to the metabolic crisis measured by brain microdialysis. In a group of patients with severe TBI, a prospective multicenter study of surface and intracortical depth combined with brain microdialysis, time-locked analysis of neurochemical responses to seizures and pseudo-periodical discharges was performed. It was found that 61% of the 34 subjects had seizures or PD, and 42.9% of the seizures were only found on the deep intracortical EEG, and in some cases lasted several hours [4]. Queiroz et al. found that changes in the excitability of neuronal networks in the hippocampus are one of the hallmarks of epilepsy; however, neuronal loss and mossy fiber sprouting are associated with enhanced inhibition rather than progressive hyperexcitability. The purpose of his research was to investigate how changes in excitability are related to spontaneous seizures expressed in DG before, during, and after seizures. For this, he used freely moving rats, and these rats developed spontaneous seizures after kainic acid-induced status epilepticus. The relationship between pulse stimulation and input-output showed that the paired pulse suppression of epilepsy patients increased, indicating that the inhibitory effect on DG during the interictal period was quite strong [5]. Florence found that the traditional diagnostic criteria for cirrhosis and renal dysfunction is a 50% increase in serum creatinine, and the final value is higher than 1.5 mg/dL, which means that patients with mild renal insufficiency have not been diagnosed and therefore have not been treated in time. In 2015, the term Acute Kidney Injury (AKI) was revised to represent acute renal dysfunction in liver cirrhosis, and it was defined as the percentage increase of 0.3 mg/dL within 48 hours, and the severity of liver cirrhosis is described by stages. Various studies in the past few years have shown that these new diagnostic criteria are effective in predicting the prognosis of patients with liver cirrhosis and AKI [6]. Gerbes found that kidney failure in cirrhosis may be caused by many reasons; although the treatment of patients with ascites and hepatorenal syndrome has been established, recent attention has been focused on acute kidney injury in cirrhosis. The reduction of central effective blood volume is the key to the pathophysiology of renal failure and ascites formation in cirrhosis, and thus he recommends infusion of albumin after massive puncture. In selected patients, transjugular intrahepatic portosystemic shunt can well control ascites and improve survival. The role of non-selective blockers in patients with cirrhosis and ascites is controversial, and AKI in cirrhosis has been redefined and has prognostic importance, and the role of renal function in patients with cirrhosis has been paid more and more attention [7]. Li et al. found that based on multimodal image data, the construction of brain tumors and their surrounding anatomical structures through fusion, three-dimensional (3D) reconstruction, and other methods can provide visual information about tumors, skulls, brains, and blood vessels for preoperative operations. He collected the computed tomography magnetic resonance imaging data of 15 patients with confirmed brain tumors. It was found that based on CT and MRI images, the entire 3D structure including tumor, brain surface, skull, and blood vessels was successfully reconstructed [8]. Li found that the Industrial Internet of Things, which connects society and industrial systems, represents a huge and hopeful paradigm shift. With the help of the Internet of Things, it is easy to collect multimodal and heterogeneous data from industrial equipment, and further analyze to discover the underlying knowledge of equipment maintenance and health. Industrial equipment fault diagnosis based on the Internet of Things data is very helpful to the sustainability and applicability of the Internet of Things ecosystem, but how to effectively use and integrate this multimodal heterogeneous data to achieve intelligent fault diagnosis is still a challenge. He proposed a new fault diagnosis method based on deep multimodal learning and fusion to solve heterogeneous data from the IoT environment where industrial equipment coexists. He designed a model by combining convolutional neural networks and stacked noise reduction automatic coding to capture more comprehensive fault knowledge and extract features from different modal data [9]. Ramachandram et al. found that a popular deep learning test platform has multimodal recognition of human activities or gestures, which involve different inputs, such as video, audio, skeletal gestures, and depth images. Deep learning architectures perform well on such problems because they can combine modal representations at different levels of nonlinear feature extraction. However, designing an optimal architecture to incorporate these learned representations is largely a nontrivial human engineering work. He regarded the fusion structure optimization as a hyperparameter search and transformed it into a discrete optimization problem under the Bayesian optimization framework. He proposed two methods to calculate the structural similarity in the search space of the tree structure of the multimodal architecture, and proved their effectiveness on two challenging multimodal human activity recognition problems [10]. Through experimental research by scholars, it is found that in recent years, the problem of epileptic seizures in patients with liver cirrhosis and overlapping HEV infection has become more and more serious. However, in their experiments, there is a lack of intelligent methods, and how to detect epileptic seizures intelligently is a difficult problem that needs to be solved today.

The innovations of this article are: (1) It introduces the related theoretical knowledge of deep multimodal fusion technology and overlapping HEV infection in liver cirrhosis, and uses the neural network algorithm to investigate and analyze the epileptic seizures of patients with overlapping HEV infection in liver cirrhosis. (2) Based on the neural network algorithm and the fusion algorithm to carry out the experiment and analysis of the epileptic seizures of patients with liver cirrhosis and HEV infection, a through investigation and analysis to prevent the epileptic seizures of patients with liver cirrhosis and HEV infection is performed.

## 2. Neural Network Algorithm Based on Deep Multimodal Learning

### 2.1. The Concept of the Neural Network Algorithm

Artificial neural networks are based on the basic principles of neural networks in biology, and after understanding the structure of the human brain and the response mechanism of external stimuli, it simulates the nervous system of the human brain based on the knowledge of network topology and sorts out complex information. In deep training, the neural network method simulates the hierarchical structure of the human brain, using the hierarchical processing process of the human neural center, such as images and sounds, and each layer extracts the features of things to establish a mapping relationship between the low-level functions and the high-level semantics of the complex. Deep learning is a kind of machine learning, and machine learning is the necessary path to realize artificial intelligence. The concept of deep learning originates from the research of artificial neural networks. Multilayer perceptron with multiple hidden layers is a kind of deep learning structure [11–13]. The deep learning structure diagram is shown in Figure 1.

As shown in Figure 1, the traditional method is to learn more useful features by building a machine learning model with many hidden layers and massive training data, so as to finally improve the accuracy of classification or prediction. Compared with traditional methods, deep learning methods usually include multiple hidden node layers, emphasizing the depth of the model structure and completing the final prediction and recognition by transforming each feature layer. Through this method, the problem of manual intervention is solved [14], and the neural network structure diagram is shown in Figure 2:

As shown in Figure 2, this article uses neural network methods to classify epileptic EEG [15].

As shown in Figure 3, due to the nonlinear and nonstationary characteristics of the EEG signal, it is difficult to directly perform data analysis on the original data, and epilepsy EEG will show typical epileptiform discharges in frequency during seizures, reflecting energy changes. This change can be used as a significant feature for judging epilepsy; therefore, converting EEG signals into spectrum signals is more conducive to feature extraction and classification of epilepsy EEG signals.

However, one problem with this model is that every time an output sequence is predicted, the decoder decodes to obtain the output sequence using the same semantic coding vector [16] as shown in Figure 4.

As shown in Figure 4, mapping high-dimensional data to a lower dimensional space solves the core problem of sparse input data, i.e., first solves the problem of high-dimensional vector space. Different semantic coding vectors are generated at each moment of the predicted output sequence, and the value *W* at the moment when the output sequence *x* is predicted is expressed by probability, as shown in:

(1) $$\begin{array}{c} W\left(x|x_{i-1},\ldots ,x_{1},y\right)=g\left(x_{i-1},w_{i},s_{i}\right). \end{array}$$

*x*_*i*−1_ is the semantic encoding vector at time *x*, and *s*_*i*_ is the summary of the hidden node state of the encoder input layer at time *x*, as shown in

(2) $$\begin{array}{c} S_{i}=\sum_{k=j}^{j-1}\alpha_{ij}H_{j}. \end{array}$$

*S*_*i*_ represents the importance of the *J*-th position in the input sequence to the *i*-th position in the output sequence, which can be a linear mapping function or a neural network, as shown in

(3) $$\begin{array}{c} \alpha_{ij}=\frac{\exp\left(e_{ij}\right)}{\sum_{k=1}^{T_{i}}\exp\left(e_{tk}\right)}. \end{array}$$

### 2.2. Convolutional Neural Network Algorithm

The most commonly used in deep learning are convolutional neural networks and recurrent neural networks [17, 18]. In the convolutional layer of a convolutional neural network, a neuron is only connected to a part of the neighboring neurons. The convolutional neural network was first applied to images, and good results were obtained in the image field. The convolutional neural network can simply learn the structural characteristics of the input data through the convolution operation of the convolution kernel, and hence it is suitable for image applications. In recent years, many medical treatment researches have also introduced convolutional neural networks and achieved good results [19–22]. The structure of the convolutional neural network can be simply divided into five layers: the input layer, convolution layer, ring layer, fully connected layer, and output layer as shown in Figure 5.

As shown in Figure 5, although the input layer is a single channel, the number of feature layers in the subsequent convolutional layer is still selected to be consistent with the image rectangle classification model. This paper believes that the depth data contain more realistic grasping features, and setting more feature layers can fully learn the grasping features [23].

Select a vector composed of the first to kth elements in the sequence S; the calculation method is as shown in

(4) $$\begin{array}{c} Q_{k}=M^{T}•S_{k-m+1}. \end{array}$$

The FULL convolution and SAME convolution process satisfy the input, the output after FULL convolution is larger than the input, and the output after SAME convolution is the same size as the input; thus, these two convolutions are again called wide convolution [24]. Since the output after VALID convolution is smaller than the input size, VAID convolution is called reverse convolution.

#### 2.2.1. Back Propagation of Convolutional Neural Network Residuals

Backpropagation is the application of gradient descent in neural networks, and the backpropagation algorithm makes neural network training possible. In the case of two-dimensional convolution, the convolution method is similar to the one-dimensional [25]method. Select a part and use the convolution kernel M to calculate the inner product, as shown in

(5) $$\begin{array}{c} Q_{ij}=≺m,s_{i-m+1}=j-n+1. \end{array}$$

After convolution, there is often a nonlinear activation function, and the nonlinear conversion of features is realized through the nonlinear function, as shown in

(6) $$\begin{array}{c} p=f\left(A+x\right). \end{array}$$

Here, *x* represents the bias voltage corresponding to the convolution kernel as a scalar, and *P* is the output of the activation function with the same magnitude as *Q* [26]. The general activation function is the sigmod function, as shown in

(7) $$\begin{array}{c} \text{sigmoid}\left(a\right)=\frac{1}{1+e^{-x}}. \end{array}$$

In order to update the network parameters, according to (5) and (6), it is only necessary to calculate the gradient of a single sample cost *δ*_*j*_^*i*^ with respect to the parameters, and for this purpose, the residual is defined as

(8) $$\begin{array}{c} \delta_{j}^{i}=\frac{\partial J_{A}\left(W,A\right)}{\partial z_{j}^{i}}. \end{array}$$

For the fully connected network, *∂J*_*A*_ represents the residual of the *j*th neuron of the lth layer, and for the convolutional layer *∂z*_*j*_^*i*^, the residual of the *j*th characteristic layer of the *l*th convolutional layer (pooling layer) is a matrix. According to the definition of residual, the residual of the neuron in the first layer of the network is derived as

(9) $$\begin{array}{c} \delta^{I}=\frac{\partial J\;{\left(W,A\right)}^{2}}{\partial z^{j+1}}=f\left(z^{i}\right). \end{array}$$

In the formula, *δ*^*I*^ means the corresponding elements are multiplied, and the residual of the current layer is defined as: the residual of the current layer is equal to the product of the connection weight of the next layer and the residual of the next layer, which is multiplied by the corresponding element of the derivative of the current layer's activation function at the weighted input of the current layer. Among them, the residual of the last layer can be determined according to the specific form and sample of the cost function [27, 28].

In the same way, assuming that the lst layer of the network is a pooling layer, the residual of the *i*-th feature layer is

(10) $$\begin{array}{c} \delta^{I}=\sum_{j=1}^{n}\delta_{ji}^{l+1}*k_{ji}^{l+1}. \end{array}$$

Once the backpropagation calculation of the residual is obtained, the gradient of the sample cost with respect to the parameters can be easily obtained, and for the fully connected network layer, as shown in

(11) $$\begin{array}{c} \frac{\partial J_{a}\left(w,a\right)}{\partial w^{i}}=\frac{\partial J_{x}\left(w,a\right)}{\partial z^{i}}. \end{array}$$

The sample cost is represented by 1; the fully connected network layer is represented by 2.

#### 2.2.2. Loss Function Based on Convolutional Neural Network

The loss function or cost function is a function that maps the value of a random event or its related random variable to a non-negative real number to represent the “risk” or “loss” of the random event. This paper uses the softmax loss function, which is in the form of adding a softmax layer at the end of the network, and is used in conjunction with the log-likelihood cost function. The softmax function is defined as shown in

(12) $$\begin{array}{c} \sigma \left(a\right)=\left\{\sigma_{1}\left(a\right),\ldots ,\sigma_{m}\left(a\right)\right\}. \end{array}$$

If a single sample a belongs to label *i*, and the output of the corresponding classification layer is *b*, then the cost on this sample is

(13) $$\begin{array}{c} a_{I=1}^{8}=\frac{\exp\left(b_{i}^{7}\right)}{\sum_{j=1}^{m}\exp\left(b_{j}^{7}\right)},\;i=1,\;m=2. \end{array}$$

Simply minimizing the cost function on the overall sample may cause the model to overfit, i.e., the model is classified better on the training data, but poorly classified on the test data. Using regularization technology can effectively avoid overfitting of the network model, as shown in

(14) $$\begin{array}{c} J\left(a,b\right)=-\frac{1}{n}\left(\sum_{j=1}^{n}\sum_{j=1}^{m}\left\{t^{\left(i\right)}=j\right\}\right). \end{array}$$

Parameter initialization: since *J*(*a*, *b*) is a nonconvex function about parameter (*a*, *b*), there are a large number of local minima. Choosing better parameters to initialize the network model can speed up the training of the network and prevent the model from falling into a local minimum. The initialization method can make the output variance of each layer of the network as consistent as possible, and the parameter initialization of the image rectangle classification model selects the Xavier method, and the initialization of the weights obeys the following uniform distribution:

(15) $$\begin{array}{c} W-N\left[-\frac{\sqrt{6}}{\sqrt{n_{j}+n_{j+1}}},\frac{\sqrt{6}}{\sqrt{n_{j}+n_{j+1}}}\right]. \end{array}$$

After the convolutional layer, in order to perform convolutional result statistics, the convolutional layer often continues. It is also called the down-sampling layer; thus, the role of the ring layer also includes one-dimensional reduction, and the commonly used rings include the largest ring, the average ring, and the random ring.

### 2.3. Recurrent Neural Network

Generally, the chain connection composed of cyclic units can be analogous to the hidden layers in feedforward neural networks, but in different discussions, the “layer” of RNN may refer to the cyclic units of a single time step or all cyclic units. Therefore, as a general introduction, the concept of recurrent neural network is introduced here [29]. In the learning process, people rely on existing knowledge, and then periodically learn new knowledge based on these foundations, and continuously increase the amount of knowledge [30]. Its general structure is shown in Figure 6:

As shown in Figure 6, because the current neural network can temporarily save the previously processed information and can be further used in the next processing, the recurrent neural network is suitable for processing time-related tasks such as sequence labeling and machine translation. The calculation method is shown in

(16) $$\begin{array}{c} s_{t}=\tanh\left(Q_{V}+Q_{S-1}\right). \end{array}$$

Both the convolutional neural network and the current neural network's parameter updates depend on the anti-attribute, and the parameters are updated by calculating the gradient. For convolutional neural networks, the gradient can be directly calculated by chain derivation rules, and depends on the current neural network. The current neural network structure can be seen as an extended chain structure, but the parameters are shared, as shown in :

(17) $$\begin{array}{c} \frac{\partial \text{Loss}}{\partial v}=\sum_{\text{i}=1}^{T}\frac{\partial \text{Loss}}{\partial v_{i}}. \end{array}$$

Assuming that the loss function is recorded as *∂*Loss, the gradient calculation formula of parameter *V* is as

(18) $$\begin{array}{c} \frac{\partial \text{Loss}}{\partial Q}=\sum_{\text{i}=1}^{T}\frac{\partial \text{Loss}}{\partial Q_{i}}. \end{array}$$

The parameters *Q* and *V* are updated according to the calculated gradient, and the more commonly used current neural networks include long-memory neural networks, short-memory neural networks, and threshold recursive units.

### 2.4. Hypergraph Fusion Algorithm Based on Multimodal Technology

#### 2.4.1. Common Hypergraph Algorithm Concepts

With the rapid development of information technology today, information exists in various forms and sources. Different forms of existence or information sources can all be called a modal, and data composed of two or more modals are called multimodal [31]. Researchers achieved the purpose of building a neural network for deep network learning by combining deep learning and multimodal data fusion [25]. In addition, the characteristics of the neural network are also found, and its advantages are used, and thus we know that the multimodal fusion model is as shown in Figure 7.

As shown in Figure 7, this method can mutually modify the data of different modalities, reflect the complementarity of multimodal data, and achieve better results. In recent years, super graphs have also been used to fuse multimodal visual features, which illustrate the nature of the image itself from various angles, and use super graphs to fuse these three characteristics together. Compared with a single visual feature, based on multimodal fusion, higher accuracy can be obtained.

#### 2.4.2. Common Hypergraph Algorithms

The hypergraph algorithm can optimally find the equivalence of the graph, and the speed is faster than the best spectrum-based peer algorithm so far. The hypergraph *δW* can be defined as

(19) $$\begin{array}{c} \delta W=\left\{e\in E|e\cap S\neq \varphi \right\}. \end{array}$$

The volume of the subset is shown in :

(20) $$\begin{array}{c} volw=\sum_{V\in W}d\left(v\right). \end{array}$$

The volume of the super-edge boundary is used to indicate the closeness of the two subsets. Then, the original optimization problem is converted into a combined optimization problem with *d* as a variable, and the optimal solution of vector *d* is equivalent to the inherent vector of the minimum eigenvalue of the constraint matrix. Therefore, the above optimization problem is a simplified solution by solving the inherent vector corresponding to the next non-negative eigenvalue that determines the smallest non-negative matrix, as shown in

(21) $$\begin{array}{c} volw=\frac{\sqrt{\partial d\;v^{-1}}}{w}. \end{array}$$

If it is a hypergraph with super edges of the same size, i.e., a homogeneous hypergraph, the results obtained are the same.

## 3. Real Epileptic Seizure Automatic Detection and Classification Recognition Experiment and Result Analysis

### 3.1. Experiment and Analysis of Epilepsy EEG Prediction Method Based on Neural Network Learning Model

In recent years, the field of artificial intelligence has developed rapidly, and more and more deep learning methods have been proposed. In addition to being widely used in image, video, audio, and other fields, these have also brought new ideas in the field of medical data and made many breakthroughs. Because the data collected from the intracranial EEG are clearer than extracranial EEG data, there are fewer interference factors, and the attenuation effect of the skull on the EEG signal is avoided. Therefore, using intracranial EEG data makes easier to determine the specific location of the epilepsy focus in the brain to facilitate the operation and prevent future epileptic seizures.

This paper mainly studies the epilepsy EEG prediction method based on the neural network learning model, and proposes a feature learning and generation method based on the deep confrontation generative neural network learning model, and analyzes and improves the model structure based on the existing model. In this paper, the use of adversarial generation network to generate data that conform to the correct data distribution enables the deep learning method to achieve better experimental results.

This article first trains and tests the combined data of 4 dogs, as shown in Figure 8:

As shown in Figure 8, Gan-Loss combined data training and testing has a maximum of 5.5% and a minimum of 1%, indicating that the trend is very unstable; S-Loss combined data training and testing has a maximum of 4.4% and a minimum of 2.1%. Although it is not very high, it is generally stable.

The experimental results prove that when all the individual data of the subjects are put together to classify, the classification effect is average. When the training progresses to about 2.2, GAN_loss drops to about 2.5, S_loss can drop to about 0.8, and the accuracy rate can reach about 58%. Because different test subjects have different shapes of seizures, seizures of various types are often accompanied by muscle contractions, limb spasms, blinking, and other actions that hinder brain waves during seizures. Each seizure pattern is very different between different test subjects, and the seizure mechanism and seizure pattern of patients are also different among multiple seizures. The mixed data experiment has a general effect, and hence the next step is to train and test each subject individually, as shown in Tables 1 and 2:

As shown in Tables 1 and 2, in order to verify the effectiveness of the method proposed in this article on a single test data, this article compares with some classic feature extraction methods. Among them, the CM feature has a very good effect on Dog D. The accuracy rate reaches 67.8%, and it has a good effect on DogB and DogC, which can reach an accuracy rate of more than 50%, but the accuracy of DogA classification is lower than 34.64%.

The first four features are feature extraction based on the original EEG signal data. The third behavior spectrum is the classification effect of the convolutional neural network, the fourth behavior spectrum is the classification result of the EFL, and the last line is the experimental result of the method, which can be seen that the experimental accuracy of this method in each epileptic seizure prediction model is very high.

### 3.2. Experiment and Analysis of Questionnaire Survey

Liver cirrhosis refers to chronic progressive liver fibrosis caused by extensive degeneration and necrosis of liver cells caused by various reasons, and its structure and blood vessel supply are destroyed; liver cirrhosis is an important reason for the increase in deaths worldwide. This article compares the trends of cirrhosis cases from 2011 to 2015, as shown in Table 3:

As shown in Table 3, the number of male cirrhosis cases has been on the rise from 2011 to 2015. In 2011, there were 1141 male cases and 989 female cases; in 2015, there were 1678 male cases and 1,290 female cases, and the number of male cirrhosis patients is significantly higher than that of females. Although the number of female cirrhosis patients is lower than that of males, it is also increasing every year. It can be known that the number of patients with liver cirrhosis increases with the growth of the year, and thus how to prevent liver cirrhosis is the most important thing at present.

This article investigates the trends of male and female cirrhosis cases from 2017 to 2018, as shown in Figure 9:

As shown in Figure 9, the growth rate of cirrhosis cases in 2017 is very unstable, and the lowest is about 5%, and the highest is about 13.5%; the growth rate of cirrhosis cases in 2018 is relatively stable, the lowest is about 10%, and the highest is about 20.5%; and the proportion of men with cirrhosis is higher than the proportion of women with cirrhosis, which is about 3% higher.

Complications such as esophageal vein tumor, gastric vein tumor rupture, infection, and hepatic encephalopathy will bring many adverse effects. In an environment with limited medical resources, patients only pay attention to hospitalization and often neglect the impact of self-health management on disease. Therefore, patients will get hospitalized repeatedly, which will increase their economic, psychological, and social burden. So far, the treatment of liver cirrhosis in China is mainly carried out in hospitals, but in order to prevent the deterioration of the liver, the treatment goal is to prevent and treat late complications. In order to increase the authenticity and reliability of the experiment, this article also investigated the etiology of cirrhosis cases in recent years, as shown in Table 4:

As shown in Table 4, the main causes of liver disease are viral hepatitis B, hepatitis B accompanied by alcoholic liver disease, alcoholic liver disease, autoimmune liver disease, and viral hepatitis C. Among them, viral hepatitis B is the most common, and viral hepatitis C is the least, and men are higher than women. Therefore, it is necessary to strengthen your body, drink less alcohol, and achieve the goal of preventing liver cirrhosis.

Different causes of chronic liver disease cause repeated degeneration and necrosis of liver cells, proliferation of fibrous tissue, and nodular regeneration of liver cells during the continuous progress of the disease. After the normal liver lobule structure is destroyed, false lobules are gradually formed, and this series of irreversible changes eventually develops into liver cirrhosis.

Cirrhosis of the liver is becoming more and more common; as each person's living environment and lifestyle and personal physique are different, the composition ratio of the main causes is also different. The main cause of liver cirrhosis in European and American countries is frequent drinking, and the primary cause of liver cirrhosis in China is hepatitis B. However, in recent years, the proportion of liver cirrhosis caused by alcohol and autoimmune factors in China has increased, which is closely related to the changes in people's lifestyle and the increase in the detection rate of autoimmune liver diseases. Generally speaking, if chronic liver disease develops to cirrhosis, it will bring many side effects, which will not only affect the quality of life of patients, but even lead to death in severe cases. Timely analysis of the causes of liver cirrhosis and the clinical characteristics of each cause plays a major role in the prevention, diagnosis, and treatment of liver cirrhosis.

Studies have found that patients with liver cirrhosis and HEV infection are more likely to suffer from epilepsy, and the frequency of seizures in this type of patients is significantly higher than that of ordinary epilepsy patients. This article investigates the frequency of epileptic seizures in patients with liver cirrhosis and overlapping HEV infection and ordinary epilepsy patients, as shown in Table 5:

As shown in Table 5, epileptic seizures of patients with liver cirrhosis and overlapping HEV infection increase with the increase in years, and the upward trend is rapid. Compared with patients with liver cirrhosis and overlapping HEV infection, the frequency of epileptic seizures in ordinary epilepsy patients is significantly lower. Therefore, it can be known that the frequency of epileptic seizures in patients with liver cirrhosis and HEV infection is significantly higher than that of ordinary epilepsy patients, and patients with liver cirrhosis are more likely to have seizures.

This article investigates the factors of epileptic seizures in patients with liver cirrhosis and HEV infection, as shown in Figure 10:

As shown in Figure 10, education level, frequency of seizures, number of medications, and depression have become important factors affecting the cognitive function of patients with epilepsy. A high degree of education, good seizure control, medications, and a healthy mental and emotional state are protective factors for improving the cognitive function of patients with epilepsy, and seizure control is one of the important factors that affects the cognitive function of patients without decline in the short term.

## 4. Discussion

In this article, related concepts such as deep multimodal fusion technology and epileptic seizures in patients with overlapping HEV infection and liver cirrhosis are described. It studied the neural network algorithm based on deep multimodal fusion technology, and explored how to analyze the epileptic seizures of patients with liver cirrhosis and overlapping HEV infection based on the neural network algorithm, and through the questionnaire survey method discussed the frequency of epileptic seizures in patients with liver cirrhosis and HEV infection, and finally expressed how to prevent liver cirrhosis.

This article investigated the prevalence factors of multiple patients with liver cirrhosis through a questionnaire survey. Finally, it was found that the main causes of liver cirrhosis were viral hepatitis B, hepatitis B combined with alcoholic liver disease, etc., among which the proportion of factors causing viral hepatitis B ranked first.

This paper also proposes a neural network algorithm based on deep multimodal fusion technology to analyze the effects of the neural network algorithm in the investigation and analysis of epileptic seizures in patients with liver cirrhosis and HEV infection.

Through the investigation, this article found that patients with liver cirrhosis are prone to seizures more frequently than ordinary epilepsy patients, and finally analyzed the cognitive factors that affect patients with epilepsy.

## 5. Conclusions

This article is mainly based on deep multimodal fusion technology, and proposes related methods of deep learning, especially neural network algorithms, which can effectively predict epileptic seizures. The theory of related knowledge such as liver cirrhosis and epileptic seizures is explained, and in the method part, not only the neural network algorithm is used, but also the data fusion model is used to achieve a brain circuit model that simulates epileptic seizures. The experimental part of this article conducted experiments on the epilepsy EEG prediction method, and found that the classification effect of the spectrogram plus convolutional neural network has a high experimental accuracy in each epileptic seizure prediction model; therefore, this method can be used to predict epileptic seizures in general medicine. Finally, a questionnaire survey was conducted on patients with liver cirrhosis, and it was found that in recent years, with the increase in patients with liver cirrhosis, more and more patients have seizures, and the frequency of seizures in patients with cirrhosis and overlapping HEV infection is higher than that of ordinary people. Therefore, in order to prevent epileptic seizures, we must first prevent and treat liver cirrhosis, and the content of this article has a certain impact on the research of epileptic seizures.

## Figures and Tables

**Figure 1:** Deep learning structure diagram.

**Figure 2:** Neural network structure diagram.

**Figure 3:** Seizure prediction model of neural network.

**Figure 4:** Coding vector prediction model.

**Figure 5:** The structure of a convolutional neural network.

**Figure 6:** Recurrent neural network structure diagram.

**Figure 7:** Multimodal fusion model based on deep network.

**Figure 8:** The GAN_loss curve of four dogs. (a) Gan-loss combined data training and testing. (b) S-loss combined data training and testing.

**Figure 9:** Comparison of trends in male and female cirrhosis cases from 2017 to 2018. (a) The trend of male and female cirrhosis cases in 2017. (b) The trend of male and female cirrhosis cases in 2018.

**Figure 10:** Factors of epileptic seizures in patients with liver cirrhosis and HEV infection. (a) Factors of epileptic seizures in patients with cirrhosis and HEV infection. (b) Factors of seizures in patients with cirrhosis and HEV infection.

**Table 1:** Five groups of canine epilepsy EEG data description.

Test subject	Interval data number	Preliminary data	Number of data channels	Sampling frequency
Dog A	400	243	15	500
Dog B	500	265	15	500
Dog C	453	276	15	500
Dog D	564	380	14	500

**Table 2:** Comparative experimental results.

Method	Dog A	Dog B	Dog C	Dog D
DCGAN + ELM	0.3464	0.5646	0.5786	0.6781
CNN	0.74	0.67	0.78	0.72
CM	0.4353	0.3532	0.3567	0.3671
SE	0.9809	0.9584	0.9367	0.5648
SRP	0.9687	0.8979	0.8732	0.8901
Splice	0.9456	0.6372	0.7853	0.5751
SS-DCGAN	0.9463	0.6854	0.7654	0.9797

**Table 3:** Trends of cirrhosis cases from 2011 to 2015.

Years	Male	Female	Total
2011	1141	989	2130
2012	1212	1097	2309
2013	1287	1108	2395
2014	1365	1201	2566
2015	1678	1290	2968

**Table 4:** Inquiry into the etiology of cirrhosis cases in recent years.

years	Male	Female	Total
Viral type B	320	229	549
Hepatitis B with alcoholic	201	200	401
Alcoholic	121	102	223
Autoimmune	109	97	206
Type C viral	45	56	101

**Table 5:** Epileptic seizure frequency survey in patients with cirrhosis and overlapping HEV infection and ordinary epilepsy patients.

Years	Patients with HEV infection (%)	Patients with common epilepsy (%)
2015	5.26	3.32
2016	6.28	4.73
2017	8.96	5.38
2018	12.31	7.80
2019	16.59	8.35

## Data Availability

The data that support the findings of this study are available from the corresponding author upon reasonable request.
